RETRACTED

# Upregulation of HYAL1 Expression in Breast Cancer Promoted Tumor Cell Proliferation, Migration, Invasion and Angiogenesis

**DOI:** 10.1371/journal.pone.0022836

**Published:** 2011-07-28

**Authors:** Jin-Xiang Tan, Xiao-Yi Wang, Xin-Liang Su, Hong-Yuan Li, Yuan Shi, Liang Wang, Guo-Sheng Ren

**Affiliations:** 1 Department of Endocrine and Breast Surgery, the First Affiliated Hospital of Chongqing Medical University, Chongqing, China; 2 Molecular Oncology and Epigenetics Laboratory, the First Affiliated Hospital of Chongqing Medical University, Chongqing, China; 3 Department of Anaesthesiology, Children's Hospital of Chongqing Medical University, Chongqing, China; 4 Department of General Surgery, the First Hospital of Jiulongpo District, Chongqing, China; Faculdade de Medicina, Universidade de São Paulo, Brazil

## Abstract

Hyaluronic acid (HA) is a component of the Extra-cellular matrix (ECM), it is closely correlated with tumor cell growth, proliferation, metastasis and angiogenesis, etc. Hyaluronidase (HAase) is a HA-degrading endoglycosidase, levels of HAase are elevated in many cancers. Hyaluronidase-1 (HYAL1) is the major tumor-derived HAase. We previously demonstrated that HYAL1 were overexpression in human breast cancer. Breast cancer cells with higher HAase expression, exhibited significantly higher invasion ability through matrigel than those cells with lower HAase expression, and knockdown of HYAL1 expression in breast cancer cells resulted in decreased cell growth, adhesion, invasion and angiogenesis. Here, to further elucidate the function of HYAL1 in breast cancer, we investigated the consequences of forcing HYAL1 expression in breast cancer cells by transfection of expression plasmid. Compared with control, HYAL1 up-regulated cells showed increased the HAase activity, and reduced the expression of HA in vitro. Meantime, upregulation of HYAL1 promoted the cell growth, migration, invasion and angiogenesis in vitro. Moreover, in nude mice model, forcing HYAL1 expression induced breast cancer cell xenograft tumor growth and angiogenesis. Interestingly, the HA expression was upregulated by forcing HYAL1 expression in vivo. These findings suggested that HYAL1-HA system is correlated with the malignant behavior of breast cancer.

## Introduction

Extra-cellular matrix (ECM) is closely correlated with tumor progression. Hyaluronic acid (HA) is a component of the ECM, it is an unsulfated anionic linear glycosaminoglycan polymer comprised of a repeating glucuronic acid and N-acetylglucosamine disaccharide motif [1]. HA keeps tissues hydrated, maintains osmotic balance and cartilage integrity [2]–[3]. HA also actively regulates cell adhesion, migration, and proliferation by interacting with specific cell surface receptors such as CD44 and RHAMM [4]. The concentration of HA is elevated in several inflammatory diseases and various carcinomas, including bladder, prostate, breast, lung, colon, and so forth [5]–[10]. Small fragments of HA, generated by Hyaluronidase (HAase), stimulate angiogenesis [11], [12]. In tumor tissues, it may promote tumor growth and metastasis probably by actively supporting tumor cell migration and offering protection against immune surveillance [13].

RETRACTED

HAases are a class of enzymes that predominantly degrade HA, they are endoglycosidases, as they degrade the β-N-acetyl-D-glucosaminidic linkages in the HA polymer [1]. HAase has been shown to alter the expression of CD44 isoforms, which may also be involved in tumor progression [14]. In addition, HAase is associated with increased tumor cell cycling [15]. The HAase levels serve as an accurate marker for detecting prostate and bladder tumors [9]–[10]. In humans, six HAase genes have been identified. Hyaluronidase-1 (HYAL1) was originally purified from human plasma and urine [16]–[17], it is the major tumor-derived HAase expressed in bladder and prostate cancer tissues, and it has characterized expression at the mRNA and protein levels in tumor cells [9], [10]. HYAL1 is a ∼55–60 kDa protein, and it is consisted with 435 amino acids. An elevated level of HYAL1 has been found in prostate, bladder, breast, head and neck cancers, etc [9]–[10], [18]–[20]. HYAL1 was the first HAase to be recognized as being expressed by tumor cells and its expression correlates with their invasive and metastatic potential [9]. No HYAL1 expression is observed in the tumor-associated stroma, although HYAL1 expression appears to correlate and perhaps induce HA production in the tumor-associated stroma [21]–[22].

Among the six HAases, HYAL1 and Hyaluronidase-2 (HYAL2) are widely distributed to degrade high molecular weight (MW) HA [23]. The HYAL2 cleaves high MW HA into ∼20 kDa HA fragments [24], which are transported intracellularly and further digested into low MW HA fragments by HYAL1 [25]. The small angiogenic HA fragments stimulate endothelial cell proliferation, adhesion and migration by activating the focal adhesion kinase and mitogen-activated protein kinase pathways [26]. HYAL1 has been found as an independent predictor of biochemical recurrence [27]. HAase levels also increase in breast cancer cells when they become metastatic [18].

We previously demonstrated that HYAL1 protein and activity were overexpression in breast cancer tissues and cells [19], [28], and breast cancer cells with higher HAase expression, exhibited significantly higher invasion ability through matrigel than those cells with lower HAase expression [28]. Knockdown of HYAL1 expression in breast cancer cells resulted in decreased cell growth, adhesion, invasion and angiogenesis [19], [29]. In this study, to further elucidate the function of HYAL1 in breast cancer, we demonstrated that forcing expression of HYAL1 in breast cancer cells promoted tumor progression in vitro and in vivo. We therefore provided functional evidence that HYAL1 is oncogenic for breast cancer and functional antagonism of HYAL1 constitutes a potential therapeutic strategy for HYAL1 positive breast cancer.

RETRACTED

## Results

### Identification of the recombinant plasmid

The HYAL1 expressing plasmids were constructed using the eukaryotic expression vector pcDNA3.1(+). The positions of the restriction enzyme digestion sites were marked (Fig. 1A). After sequence analysis, transfection of the recombinant plasmid pcDNA3.1-HYAL1 or pcDNA3.1 empty vector into MCF7 cells, respectively. After stably transfected cells were individually selected, the HYAL1, HYAL2 and the housekeeping gene β-actin mRNA levels were measured using RT-PCR. Compared with the control group, the pcDNA3.1-HYAL1 transcripts were sharply up-regulated (Fig. 1B). Accordingly, HYAL1 protein levels were increased in pcDNA3.1-HYAL1 transfected cells too, as indicated by western blotting (Fig. 1C) and immunofluorescence (Fig. 1D) analyses. The pcDNA3.1 empty vector did not substantial affect the endogenous HYAL1 expression, and there was no difference in the HYAL2 expression among groups. These results demonstrated that pcDNA3.1-HYAL1 was up-regulated specifically and effectively.

**Figure 1:** Identification of the recombinant plasmid. Construction of the recombinant eukaryotic expression vector pcDNA3.1(+) containing the HYAL1 gene used in the studies. The positions of the restriction enzyme digestion sites were marked (A). Transfection of the recombinant plasmid pcDNA3.1-HYAL1 or pcDNA3.1 empty vector into MCF7 cells, respectively. RT-PCR (B), Western blot (C) and immunofluorescence (D) analysis validated the successful transfection and the expression of the HYAL1 mRNA and protein were up-regulated in pcDNA3.1-HYAL1, the pcDNA3.1-HYAL1 did not substantially affect the HYAL2 expession.

### Upregulation of HYAL1 in breast cancer cells increased colony formation and enhanced cell proliferation

To determine the functional consequences of forcing HYAL1 expression in human breast cancer cells, we generated the breast cancer cell lines MCF7 and ZR-75-30 with upregulation of HYAL1 by stable transfection with HYAL1 expression vector (termed MCF7-HYAL1 and ZR-HYAL1) or the empty pcDNA3.1 vector (designated MCF7-Vec and ZR-Vec), respectively. Soft agar assays were then performed to determine whether upregulation of HYAL1 could enhance colony formation in an anchorage-independent culture system. In soft agar assays, the number of colonies of MCF7-HYAL1 and ZR-HYAL1 were 42.2±4.6 and 34.9±4.8, however, the number of colonies of MCF7-Vec and ZR-Vec were 31.1±5.4 and 26.2±3.6, respectively. There was a statistically significant increase in the number of colonies of pcDNA3.1-HYAL1 compared to pcDNA3.1-Vec control cells (Fig. 2A; *p*<0.01). In 3D Matrigel cultures, the size (µm) of colonies of MCF7-HYAL1 (53.2±16.0) and ZR-HYAL1 (48.8±21.5) were bigger than MCF7-Vec (38.3±12.8) and ZR-Vec (39.1±10.9), respectively (Fig. 2B; *p*<0.05). Then, we examined the proliferation activity of the transfected cells using MTT assay. As shown in Fig. 2C, compared with the controls, the proliferation rates of MCF7-HYAL1 and ZR-HYAL1 transfected cells were increased significantly (*p*<0.01). These results indicated that HYAL1 is correlated with cell proliferation.

RETRACTED

**Figure 2:** Upregulation of HYAL1 in breast cancer cells increased colony formation and enhanced cell proliferation. MCF7-HYAL1 and ZR-HYAL1 enhanced the number of colony formation in Soft agar (A) and size of colony in 3D Matrigel (B) (*p*<0.01, *p*<0.05, respectively), (original magnification ×100). MTT assay showed that MCF7-HYAL1 and ZR-HYAL1 increased cell proliferation rates (C; *p*<0.01).

### Upregulation of HYAL1 expression increased HAase activity, and reduced HA expression

HAase ELISA-like assay was carried out as described previously. As shown in Fig.3A, the amount HAase activity (mU/mg) in MCF7-HYAL1 (14.78±2.59) and ZR-HYAL1 (12.69±2.78) were higher than MCF-Vec (5.34±1.07) and ZR-Vec (4.60±1.09), respectively (*p*<0.01). However, compare with MCF-Vec (0.50±0.10) and ZR-Vec (0.43±0.11), the HA levels (µg/mg) in MCF7-HYAL1 (0.35±0.09) and ZR-HYAL1 (0.26±0.08) were decreased, respectively (Fig.3B; *p*<0.05). These results demonstrated that pcDNA3.1-HYAL1 can enhance the HAase activity, and the HYAL1 could degrade HA.

**Figure 3:** Summary of HAase activity and HA expression by ELISA-like assay. In MCF7 and ZR-75-30 cells, the HAase activity was increased significantly by pcDNA3.1-HYAL1 transfectants (A; *p*<0.01). However, the HA expression was decreased (B; *p*<0.05).

### Upregulation of HYAL1 expression promoted breast cancer cell cycling

To determine whether HYAL1 regulates cell cycle progression induced by growth factor, Flow cytometry was performed to analyze cell cycle phases. Compared with MCF7-Vec and ZR-Vec, both in MCF7-HYAL1 (Fig. 4A) and ZR-HYAL1 (Fig. 4B) transfectants, the number of cells in G_0_/G_1_ phase were decreased, but those in S phase were increased (*p*<0.05, *p*<0.01, respectively). No alterations in G_2_/M phase were observed (*p*>0.05). These results indicated that HYAL1 is correlated with cell cycle in vitro.

RETRACTED

**Figure 4:** Upregulation of HYAL1 effected on cell cycle. The MCF7-HYAL1 (A) and ZR-HYAL1 (B) transfectants had a higher portion in S phase and a lower portion in G_0_/G_1_ phase ((*p*<0.05, *p*<0.01, respectively)). No alterations in G_2_/M phase were observed (*p*>0.05).

### Upregulation of HYAL1 expression enhanced the cell migration, invasion and angiogenesis potential of breast cancer cells

One of the most distinct features of breast cancer cell is the invasive growth pattern and promotion in angiogenesis, which prevents total surgical resection. Therefore, we evaluated the effect of HYAL1 upregulation on cell migration, invasion and angiogenesis properties.

To study the effect of HYAL1 upregulation on the cell migration, wound-healing assays were carried out by allowing the cells to move to the scar region for 24 h and 48 h. We observed that forced expression of HYAL1 in both MCF7 and ZR-75-30 cells did indeed stimulate wound closure compared with their respective vector-transfected cells (Fig. 5A and B; *p*<0.05, *p*<0.01, respectively).

**Figure 5:** Upregulation of HYAL1 in breast cancer cells promoted cells migration in vitro. The MCF7-HYAL1 (A) and ZR-HYAL1 (B) transfectants promoted wound closure compared with their respective empty vector transfected cells (*p*<0.05, *p*<0.01, respectively), (original magnification ×100).

Invasion assays were performed using ECM gel-coated transwell culture chambers. After 48 h of incubation, invading cells were counted. We observed that forced expression of HYAL1 in both MCF7 and ZR-75-30 cells did indeed stimulate cell invasion compared their respective vector-transfected cells (Fig. 6A; *p*<0.01). The potential of promoting angiogenesis was analysed by in vitro angiogenesis assay. CRL-1730 cells formed branch-like or net-like structures when co-cultured with MCF7 and ZR-75-30 cells, which were not seen in the absence of tumor cells. The numbers of branch-like and net-like structures formed by CRL-1730 co-cultured with MCF7 cells were acutely increased in the MCF7-HYAL1. Similarly, in the ZR-75-30 and CRL-1730 co-culture system, compared with ZR-Vec, the numbers of branch-like and net-like structures in ZR-HYAL1 group was increased obviously. (Fig. 6B; *p*<0.05). These results demonstrated that HYAL1 is correlated with cell migration, invasion and angiogenesis potential of breast cancer cells.

**Figure 6:** Upregulation of HYAL1 in breast cancer cells promoted cell invasion and angiogenic capability in vitro. Invasion assays (A) were performed using ECM gel-coated transwell culture chambers. 48 h after seeding for both MCF7 and ZR-75-30, the number of invasive cells was increased in pcDNA3.1-HYAL1 transfectants (*p*<0.01). Angiogenesis assay (B) for CRL-1730 cells formed branch-like or net-like structures through co-culture with MCF7 and ZR-75-30 cells. After 96 h co-culture, the number of vessels developed by CRL-1730 cells was enhanced in pcDNA3.1-HYAL1 transfectants (*p*<0.05), (original magnification ×100).

RETRACTED

### Upregulation of HYAL1 expression promoted the tumorigenesis of breast cancer cells in vivo

To evaluate the tumorigenetic capability of HYAL1 upregulation tumor cells in vivo, 20 mice were injected into the mammary fat-pad with 1×10^7^ MCF7 cells, and the tumor growth was monitored for a period of 9 weeks. These mice were randomly divided into 2 groups (MCF7-Vec and MCF7-HYAL1) with 10 mice in each group. All of mice developed tumors at the end of the experiment. However, the mice treated with MCF7-HYAL1 cells showed a significant enhancement of tumor growth compared with those treated with MCF7-Vec cells (Fig. 7A; *p*<0.01). 9 weeks after inoculation, the average tumor weight in MCF7-HYAL1 (3.18±0.64 g) was heavier than MCF7-Vec (1.91±0.49 g) (Fig. 7B; *p*<0.01). Western blot (Fig. 7C) and immunohistochemistry (Fig. 7D) analysis confirmed that the HYAL1 protein expression was significant enhanced in the MCF7-HYAL1 group. The HYAL2 was not changed obviously. Ki67 is a molecular maker that is related to proliferation, was located in the nucleus. Compared with MCF7-Vec, the ki67 was highly expressed in MCF7-HYAL1 group (Fig. 7D). CD31 is an endothelial marker, so the microvessel density (MVD) of the tumor tissue was assessed by CD31 immunohistochemistry analysis. Compared with MCF7-Vec, the expression of CD31 in MCF7-HYAL1 was increased obviously (Fig. 7D). In addition, compared with MCF7-Vec (7.26±1.56) group, the HAase activity (mU/mg) in the MCF7-HYAL1 (18.42±3.23) group was enhanced significantly (Fig. 7E; *p*<0.01). At same time, the HA expression level (µg/mg) in MCF7-HYAL1 (15.69±3.63) was higher than MCF7-Vec (11.75±2.21) (Fig. 7F; *p*<0.05). These data indicated that HYAL1 could promote tumor proliferation and angiogenesis in vivo, and the HA expression was increased in tumor tissue during enhancing tumor malignant potentiality, although the HYAL1 could degrade HA.

**Figure 7:** Upregulation of HYAL1 increased tumor growth, angiogenesis, HAase activity and HA expression of MCF7 cells in vivo. Representative mouse bearing tumors, the average tumor volume (A) from 5^th^ weeks and tumor weight (B) in MCF7-HYAL1 group were increased significantly than in MCF7-Vec group (*p*<0.01). Western blot (C) and immunohistochemistry (D) analysis showed that the expression of HYAL1 protein was enhanced in the MCF7-HYAL1 group obviously, but HYAL2 levels were not altered. Compared with MCF7-Vec, expression of ki67 and CD31 were increased in MCF7-HYAL1 (D). ELISA-like assay measured HAase activity (E) and HA levels (F) present in the tissue extracts, the HAase activity and HA levels in MCF7-HYAL1 were higher than MCF7-Vec (*p*<0.01, *p*<0.05, respectively).

RETRACTED

## Discussion

In this study, the eukaryotic expression plasmid pcDNA3.1-HYAL1 was constructed to force HYAL1 expression in breast cancer cell lines MCF7 and ZR-75-30. Our results showed that upregulation of HYAL1 resulted in cell growth increase in vitro and in vivo (Fig. 2, 7A and 7B). It was also identified that HYAL1 expression in bladder cells regulated tumor gowth [22]. These results suggested that HYAL1 expression in tumor cells is required for cell proliferation. Meanwhile, upregulation of HYAL1 expression enhanced the proportion of cells cycling in S phase (Fig. 4), which is consistent with Lin et al. [15] and our previous researches [19], [29]. Based on the analysis of cell cycle regulators, HYAL1 affects cell proliferation probably by regulating cell cycle.

Our finding that upregulation of HYAL1 in breast cancer cells could enhance the HAase activity significantly (Fig. 3A), and the HA expression was decreased obviously (Fig. 3A) in vitro, these results identified that HYAL1 could degrade HA. Which was according with previous researches [19], [25]. Interestingly, upregulation of HYAL1 expression enhanced the HAase activity (Fig. 7E), at the same time, the HA expression was increased (Fig. 7F) in vivo. Lokeshwar et al. [22] found that high level of HA was expression in tumor-associated stroma of HYAL1-sense tumor specimen, but very low HA expression was observed in the stromal compartment of HYAL1-antisense tumor specimens. Which indicated the HYAL1 could induce the stroma cells of tumor to secrete HA, although it could cleave HA.

In addition to the effect of HYAL1 on tumor growth, its effects on tumor cell migration and invasion are interesting. Our previous researches showed that breast cancer cells with higher HAase expression, exhibit significantly higher invation ability through matrigel than those cells with lower HAase expression [28]. Knockdown of HYAL1 expression in breast cancer cells resulted in decreased cell invasion [19]. HYAL1 was also an independent prognostic indicator for predicting biochemical recurrence in prostate cancer and increased metastatic potential in a prostate cancer model [27]. In the current study, we demonstrated that upregulation of HYAL1 expression in MCF7 and ZR-75-30 cells resulted in high metastasis potential and altered several functions such as cell migration and invasion in vitro (Fig. 5 and 6A). These observations suggested that HYAL1 plays a role in promoting the invasive potential of breast cancer cells. It might also be a marker predicting subsequent development of invasive breast cancer.

RETRACTED

One of the well-studied functions of the HA and HAase system is the generation of angiogenic HA fragments [30]. These angiogenic HA fragments have been shown to induce endothelial cell proliferation, migration, and adhesion [26], [31]. The secretion of HAase by tumor cells has been shown to induce angiogenesis [32]. Angiogenic HA fragments are present in the urine of grade 2 and 3 bladder cancer patients, suggesting that the HA and HYAL1 system is active in bladder cancer [33]. The HYAL1 and HYAL2 are widely distributed and degrade high MW HA in collaboration with CD44 [23]. We previously demonstrated that knockdown of HYAL1 expression in breast cancer cells resulted in decreased angiogenesis [19]. In this study, we showed that upregulation of HYAL1 expression induced higher angiogenesis in vitro and in vivo (Fig. 6B and 7D). This was in accordance with previous reports that HYAL1 over-expression increased MVD in rat colon carcinoma xenografts [34], as well as the correlation of HYAL1 with MVD in bladder tumor [22]. Which suggests that HYAL1 promotes tumor angiogenesis might be a general effect. Further studies characterizing this in other cancer models would be interest.

At present, whether HAase is a tumor promoter or a repressor has been controversial. The results presented in this study showed that forcing HYAL1 expression promoted tumor growth, invasion and angiogenesis supporting its role as a tumor promoter. HYAL1 levels in various cancers were associated with high-grade invasive tumors [9]–[10], [20], [27]. However, Jacobson et al. [34] found that the overexpression of HYAL1 by cDNA transfection in a rat colon carcinoma line decreased tumor growth, although the tumors were angiogenic. HYAL1 and HYAL2 have been identified to inhibit lung and renal carcinoma cell growth in vivo but not in vitro [35]. Nykopp TK, et al found that HYAL1 and HYAL2 were coexpressed and significantly downregulated in endometrioid endometrial cancer and correlated with the accumulation of HA [36]. The controversy surrounding HAase as a tumor promoter or a suppressor was recently explained by Lokeshwar et al [1], [21]. Selection of cells for expression of different HYAL1 levels showed that cells expressing amounts found in tumor tissues and cells promote tumor growth, invasion and angiogenesis. In contrast, cells with HAase levels exceeding 100 milliunits/10^6^ cells, (i.e.; levels that are not naturally expressed by tumor cells) exhibit reduced tumor incidence and growth due to induction of apoptosis. Therefore, the function of HAase as a tumor promoter or a suppressor is a concentration dependent phenomenon and levels in genitourinary tumors are consistent with tumor cell derived HAase acting mainly as a tumor promoter.

RETRACTED

It is also noteworthy that other proteins related to HA synthase (HAS) and HA-receptor CD44 and RHAMM are also involved in tumor growth and metastasis. For example, overexpression of HAS2, HYAL2 and CD44 is implicated in the invasiveness of breast cancer [37]. Blocking HAS3 expression in prostate cancer cells decreased cell growth in vitro and tumor growth in vivo [38]. Silencing of HAS2 suppressed the malignant phenotype of invasive breast cancer cells [39]. HAS2 expression induced mesenchymal and transformed properties in normal epithelial cells, but interestingly, HAS2 expression in the absence of HAase decreased tumor growth in glioma cells. Moreover, interaction between RHAMM and HA fragments was known to induce the mitogen-activated protein kinase pathway, and over-expression of RHAMM was a useful prognostic indicator for breast cancer [40]. Down-regulated CD44 and HA synthase while upregulating the HAases, suggested that dynamic feedback signalling and complex mechanisms occur in the net deposition of HA [41]. These results showed that the HAS-HA-HAase system is involved in the regulation of tumor growth and invasion.

Summarizing the observations by us and others, we favor the hypothesis that HYAL1 may play a critical role in the longevity of a wide spectrum of breast cancer cells. In our study, upregulation of HYAL1 promoted the cell growth, migration, invasion and angiogenesis. Interestingly, forcing HYAL1 expression induced stoma cells of tumor to secrete HA in vivo, although HYAL1 could cleave HA. To date the expression pattern and function of the HYAL1 gene in human tumors are not completely elucidated. As to the mechanism of how HAS-HA-HAase system influences the biology characteristics of human breast cancer cells, more investigations will be accomplished in the future.

## Materials and Methods

### Cell lines and cell culture

The human breast cancer cell lines MCF7 and ZR-75-30, mouse embryonal fibroblast cell line HIH-3T3 and human umbilical vein endothelial cell line CRL-1730 were acquired from the cell bank of Shanghai Institute of Biological Sciences, Chinese Academy of Sciences. These cells were maintained with RPMI1640 medium (Gibco BRL), supplemented with 10% (v/v) fetal bovine serum (FBS) (Gibco BRL). The medium was replaced every 2 d, cells were passaged every 5 to 6 d, checked routinely and cultivated in a 5% (v/v) CO_2_ incubator at 37°C.

RETRACTED

### Plasmid construction and transfection

Total RNA was extracted from breast cancer cells using a RNA extraction kit (Invitrogen). Total RNA (∼1 µg) was subjected to first strand cDNA synthesis using a Superscript*™* pre-amplification system and oligo(dT) primers (Invitrogen). The PCR primers for the entire coding region of HYAL1 (611-1918) designed with HYAL1 cDNA sequence (Genebank: U96078), the forward primer was 5′-GAGAAGCTTGCCGCCATGGCAGCCCACCTGCTTCCC-3′, the reverse primer was 5′-CAATTGTCACCACATGCTCTTCCGCTCACACCA-3′. PCR conditions were as follows: 4 min for pre-denaturation at 94°C, then 94°C for 15 s, 55°C for 15 s and 72°C for 30 s for 30 cycles, and a final extension at 72°C for 10 min. The PCR product (1300 bp) was purified and restrictively digested with Hind III and Mfe I, the plasmid pcDNA3.1(+) (Invitrogen) was purified and restrictively digested with Hind III and EcoR I, then cloned the PCR product into pcDNA3.1 to form pcDNA3.1-HYAL1, the pcDNA3.1 vector was treated as a control.

For transfection, MCF7 and ZR-75-30 were seeded in six-well plates at 5×10^5^/well and incubated in 5% CO_2_ 95% air incubator at 37°C. When cells were ∼70% confluence, cells were transfected with Lipofectamine 2000 (Invitrogen) transfection reagent according to the manufacturer's protocol. Recombinant plasmid (4 µg) were mixed with Lipofectamine and pre-incubated for 20 min at room temperature in serum-free and antibiotic-free RPMI1640. MCF7 cells transfected with pcDNA3.1-HYAL1 and pcDNA3.1 vector were named as MCF7-HYAL1 and MCF7-Vec, ZR-75-30 cells transfected with pcDNA3.1-HYAL1 and pcDNA3.1 vector were named as ZR-HYAL1 and ZR-Vec, respectively. G418 (500 µg/µl) was applied to stable screeing and isolating the resistant colonies. At the same time, corresponding empty vector was transfected as control.

### Semi-quantitative reverse transcription-polymerase chain reaction (RT-PCR)

Total RNA extraction was same as before, following manufacturer's instructions. The reverse transcription was carried out with a SuperScript first-strand synthesis system (Invitrogen) using Oligo(dT)_12-18_ primers. cDNA was amplified by Taq DNA polymerase (Promega, USA). Human β-actin gene was used as an internal control. Each PCR program involved a initial step denaturation 5 min at 94°C, followed by 28 cycles (for HYAL1, HYAL2 and β-actin) at 94°C for 20 s, 62°C for 20 s and 72°C for 30 s, at last 72°C for 10 min. DNA primer sequences were designed as follows: for human HYAL1 gene (Accession No. U96078), Sense: 5′-TGGATGGCAGGCACCCTCCA-3′, and antisense strand: 5′-CACCAGCAGCCACAGCCACA-3′, the amplicon size is 289 bp. For human HYAL2 gene (Accession No. U09577), Sense: 5′-TGGCCCGCAATGACCAGCTG-3′, and antisense strand: 5′-GCCGCACTCTCGCCAATGGT-3′, the amplicon size is 262 bp. For β-actin gene (accession No. NM_001101), sense: 5′-AAATCTGGCACCACACCTTC-3′, reverse primer, 5′-GGGGTGTTGAAGGTCTCAAA-3′, the amplicon size was 139 bp. The PCR amplified products were separated by 1.5% agarose gels electrophoresis, and the bands were visualized by staining with 0.5% Goldview. Gel images were obtained and the densities of PCR products were quantified by using densitometry methods.

RETRACTED

### Western blot analysis

The cells and fresh tissue specimens (0.5–1 g) were harvested and total protein was extracted with RIPA buffer containing protease inhibitors, protein concentration was determined by the Bradford assay (Bio-Rad Laboratories, Hercules, CA). Equal amounts of protein were subjected to 7.5% SDS–polyacrylamide gel and the resolved proteins were transferred electrophoretically to PVDF membranes (Millipore, Bedford, MA, USA). Membranes were blocked for 1 h with 5% non-fat milk in PBST buffer at room temperature, then were incubated with antibodies against HYAL1 (rabbit polyclonal; 1∶500; Sigma, USA), HYAL2 (rabbit polyclonal; 1∶500; Abcam, UK), and β-actin (rabbit polyclonal; 1∶1000; Santa Cruz, CA) for overnight at 4°C, respectively. The membranes were washed for three times with PBST, and then were incubated with the respective secondary antibodies for 1 h at room temperature. Membranes were incubated with enhanced chemiluminescence (ECL) (Pierce, Rockford, IL, USA), exposed to X-ray film for 1–2 min. The results were analyzed by using the Quantity One 4.6.3 software (Bio-Rad, Hercules, CA).

### Immunofluorescence

The transfected cells were cultured on sterile cover slips for 24 h and washed twice with cool PBS. Cells were then fixed with 2% formaldehyde, permeabilized with 0.1% Triton X-100, blocked with 2% BSA for 30 min at room temperature, and incubated with the primary antibody overnight at 4°C. Samples were washed, incubated with the secondary antibody for 30 min. Immunofluorescence was analysed using a confocal microscope.

### Soft agar growth assay

pcDNA3.1-Vec or pcDNA3.1-HYAL1 transfected cells (0.5×10^5^ cells/well in 6-well plate) were suspended in 3 ml RPMI1640 containing 10% FBS (pre-warmed to 37°C), and 300 µl of 3% agarose in PBS (pre-warmed to 60°C) was added. Agar suspended cells (1 ml/well in 6-well plates) were plated out in dishes coated with 1 ml of agar-coated dishes (0.6% agarose in RPMI1640). After solidification at room temperature for 20 min, 3 ml complete medium was added to each well and cells were incubated at 37°C in a humidified atmosphere of 5% CO_2_ (v/v) in air for 2 weeks. After this period, 10 fields were randomly selected and the numbers of colony were counted under a microscope.

RETRACTED

### 3D Matrigel culture

Matrigel basement membrane matrix (BD Biosciences, San Jose, CA) was thawed on ice and coated onto 24-wells cluster plates as a bottom layer. Subsequently, a total of 5,000 cells in 100 µl growth medium resuspended with 100 µl Matrigel was seeded on top of this bottom layer. Growth medium (0.5 ml) was added on top of the Matrigel after the polymerization was completed. Experiments were performed in triplicate. After 10 days, colonies were counted and colony sizes were measured under the stereomicroscope at 100× magnification.

### MTT proliferation assay

The capability of cell proliferation was measured by [3-(4, 5-dimethylthiazol-2-yl)-2, 5-diphenyltetrazolium bromide] MTT assay. Briefly, cells were plated at 5×10^3^ cells/well in 96-well plates and incubated for 0, 2, 4, 6, 8 and 10 d, respectively. Then cells were incubated with 20 µl MTT (10 mg/ml) for 4 h at 37°C and 100 µl DMSO (Sigma Chemical Co., USA) was pipetted to solubilize the crystal product for 10 min at room temperature. The absorbance (A) of each well was measured with a microplate reader (Bio-Rad) at a wavelength of 490 nm. This experiment was repeated three times.

### ELISA-like assay for HAase activity

HAase activity in serum-free conditioned medium of transfectants was assayed using the HAase ELISA-like assay as described previously [19]. Fresh tissue specimens (∼0.5–l.0 g) were suspended in an ice-cold homogenization buffer (5 mM Hepes pH 7.2 and 1 mM benzamidine-HCl) and homogenized for 30 s using the tissue homogenizer. The tissue extracts were clarified by centrifugation at 10,000 rpm for 30 min. The extracts were assayed for protein concentration, HAase activity and HA expression.

### ELISA-like assay for HA

The HA ELISA-like assay was described previously [19]. Briefly, ELISA plates coated with HA binding protein were incubated with samples or standards (1 h, room temperature) in triplicate, washed four times with washing buffer, incubated with a solution containing horseradish peroxidase-conjugated HA-binding protein (30 min, room temperature), washed again four times, and incubated with 100 µl of the substrate solution in the dark at room temperature. After 30 min, the reaction was stopped by adding 50 µl stop solution to each well, and the absorbance was measured at a wavelength of 405 nm.

### Flow cytometry assay

Different cell cycle phases (G_0_/G_1_, S and G_2_/M phase) are characterized by different DNA contents. The control, pcDNA3.1-Vec and pcDNA3.1-HYAL1 transfected cells were harvested with trypsin-EDTA, washed with chilled PBS twice and fixed with 70% ethanol at −20°C for 2 h, respectively. The fixed cells were pelleted, re-suspended in PI/RNase/PBS (100 µg/ml propidium iodide and 10 µg/ml RNase A) for at least 30 min at 37°C in dark. Cell cycle analysis was performed on flow cytometer. This experiment was repeated three times.

RETRACTED

### Wound healing assay

Cells were cultured in standard conditions, as described above. Until 100% confluence, the migration potency was determined using scratch wound healing assay. The scratched plates were photographed at the center of the wells using a standard magnification of 100×. The scratched cells were maintained under standard conditions for 24 hr and 48 hr. Plates were washed once again, and then the plates were photographed at the same sites of the wells using the same magnification. The cells migrating into the scratched area from the wound edge per picture were counted. The impact of pcDNA3.1-HYAL1 on cell migration potency was evaluated by comparing the mean of migration width with pcDNA3.1 empty vector.

### Cell invasion assay

Invasion capability in vitro was measured in transwell chambers (Costar Inc, USA) according to the protocol of the manufacturer. Briefly, the upper chambers of the transwell inserts were coated with 100 µl diluted ECM gel solution at 37°C for 4 h, and then pretreated with serum-free RPMI1640 medium at 37°C for 1 h before seeding the breast cancer cells at a density of 1×10^5^/well in 100 µl medium with 1% FBS. The lower chambers were filled with 500 µl RPMI1640 with 10% FBS and HIH-3T3 contained medium as a chemoattractant. The transwells were then incubated at 37°C with 5% CO_2_ for 48 h to allow cells to migrate. At the end of incubation, the cells on the upper side of the insert filter were completely removed by wiping with cotton swab, and the cells that had invaded through the ECM gel-coated filter were fixed in ethanol and stained with H&E. For quantification, the cells were counted under a microscope on 5 random fields at 100×. This experiment was repeated three times.

### Angiogenesis assay

Human umbilical vein endothelial cell line CRL-1730 were allowed to grow in transwell chambers coated with ECM gel as described above for the invasion assay (2×10^5^ cells/chamber). At the same time, the breast cancer cells were plated into 6-well plates (2×10^5^ cells/well), and cultured overnight. Then the transwell chambers were set in the 6-well plates where tumor cells were already added. The cells were co-cultured for 96 h, and the medium was changed every 24 h. The transwell chambers were washed three times with PBS, fixed in ethanol and stained with H&E. The membranes were carefully taken out of the chamber, set on glass slides, covered with a coverslip, observed under microscope, and documented with a digital imaging system (Leica MD20, Germany). The degree of angiogenesis was measured by the following method: number of branch points and the total number of branches per point, with the product indicating the degree of angiogenesis. This experiment was repeated three times.

RETRACTED

### In vivo assay

Balb/c nude mice were purchased from Vital River Lab Animal Technology Co. Ltd, and maintained under specific-pathogen-free conditions in Experimental Animal Department of the Chongqing Medical University (Chongqing, China). The protocols were approved by the Institutional Animal Care and Use Committee in Chongqing Medical University (CQMU-2008-127). Mice were randomly divided into 2 groups (MCF7-Vec and MCF7-HYAL1) with 10 mice in each group. MCF7 cells at 1×10^7^ cells per l00 µl of serum-free medium were injected orthotopically into the mammary fat-pad of 6 weeks old female Balb/C nude mice. Tumor diameters were measured one time per week with a caliper, and the volume of tumors were calculated by the following formula: x × y^2^/2, where x is the largest diameter of the tumor and y is the shortest diameter. At 9^th^ week after the injection, the tumors were harvested for western blot, immunohistochmistry, HAase activity and HA levels analysis.

### Immunohistochemistry staining

The tissue sections (∼5 µm) were de-paraffinized in xylene, rehydrated in graded ethanol solutions, permeabilized in 0.1% Triton X-100 and 0.1% sodium citrate. The endogenous peroxidase activity was quenched by incubation of the sections in 0.3% hydrogen peroxide with methanol. Subsequently, the slides were treated with 1% bovine serum albumin for 30 min to reduce nonspecific binding, followed by incubation overnight with antibody against HYAL1 (rabbit polyclonal; Sigma, USA), HYAL2 (rabbit polyclonal; Abcam, UK), Ki67 (rabbit polyclonal; Abcam, UK) and CD31 (rabbit polyclonal; Abcam, UK) at a dilution of 1∶200, respectively. After washing, the slides were further incubated with HRP-conjugated secondary antibody followed by 3,3-diaminobenzidine solution at 4°C for 30 min. Hematoxylin was used for nucleus counterstaining. For negative controls, the antibody was replaced by normal goat serum. Slides were photographed with microscope attached with CCD camera.

### Statistical analysis

Results are represented as means ± standard deviation (SD). Paired and 2-tailed Student's t-tests were used to compare results from the experiments. A *p*-value of less than 0.05 was considered statistically significant.
